The article "Effect of whole-body cryotherapy treatments on blood morphology and blood rheology: red blood cell deformability, red blood cell aggregation in healthy subjects" was published in 2023. Journal: Clin Hemorheol Microcirc.

# Effect of whole-body cryotherapy treatments on blood morphology and blood rheology: red blood cell deformability, red blood cell aggregation in healthy subjects

**DOI:** 10.3233/CH-221658

**Published:** 2023-04-07

**Authors:** Bartłomiej Ptaszek, Szymon Podsiadło, Aneta Teległów

**Affiliations:** a Institute of Applied Sciences, University of Physical Education in Krakow, Krakow, Poland; b Institute of Clinical Rehabilitation, University of Physical Education in Krakow, Krakow, Poland; c Institute of Basic Sciences, University of Physical Education in Krakow, Krakow, Poland

**Keywords:** whole-body cryotherapy, blood morphology, blood rheology, red blood cell deformability, red blood cell aggregation

## Abstract

**OBJECTIVE:**

assessment of the effect of a series of 20 whole-body cryotherapy sessions on the morphological and rheological indicators of blood in healthy people.

**METHODS:**

The experimental group consisted of 15 women and 15 men who underwent a series of whole-body cryotherapy treatments. The control group consisted of 15 women and 15 men - without intervention. For the analysis of blood biochemical parameters, venous blood was collected twice: Study 1: on the day of the commencement of whole body cryotherapy / from the control group; and Study 2: after a series of 20 cryotherapy sessions / from the control group (4 weeks).

**RESULTS:**

After whole-body cryotherapy a statistically significant decrease in RBC, HGB, HCT, MCV, EI 0.30 and an increase in MCHC and EI 2.19–60.30 were observed in women, as well as a decrease in MCV, MCH, AI and an increase in PLT, EI 0.30–60.30, AMP, T1/2 in men.

**CONCLUSIONS:**

The use of whole-body cryotherapy causes changes in blood counts in various directions and has a positive effect on the rheological properties of blood in women and men - it increases the elongation index and reduces the aggregation index.

## 1 Introduction

Whole body cryotherapy (WBC) is used to induce physiological, local, and general defense responses that help restore and maintain homeostasis. Cryotherapy is used to reduce pain and inflammation. The use of cold also reduces swelling and muscle tension, and increases muscle strength and joint mobility. Improvement in metabolism and well-being is also observed. The body’s response to WBC involves changes in many systems: the immune, endocrine, vascular, and muscular systems and nervous [1–3]. Many respondents proved the relationship between the use of cold in therapy and changes in the level of certain enzymes and hormones [1, 4–7].

Red blood cell deformability is of great importance in the flow of blood cells through capillaries of a very small diameter (smaller than these cells) [8–10]. There are many reasons for the decline in these efficiency: disease factors, mechanical damage and, above all, the aging of the organism. The phenomenon of red blood cell aggregation is a physiological and reversible phenomenon that plays an important role in blood flow at low shear rates and significantly increases blood viscosity and plasma viscosity determines the perfusion of microvessels [8, 11, 12].

The article "Effect of whole-body cryotherapy treatments on blood morphology and blood rheology: red blood cell deformability, red blood cell aggregation in healthy subjects" was published in 2023. Journal: Clin Hemorheol Microcirc.

The aim: assessment of the effect of a series of 20 whole-body cryotherapy sessions on the morphological and rheological indicators of blood in healthy people.

## 2 Material and methods

### 2.1 Participant characteristics

The presented prospective, controlled study followed the tenets of the Declaration of Helsinki, was approved by the Bioethical Commission of the Regional Medical Chamber in Krakow (approval No. 194/KBL/OIL/2019 of 17/09/2019). Overall, 77 people applied to the study, and 60 were finally selected to participate in the research program. The qualification for the tests was conducted by a rehabilitation doctor and a physiotherapist (health assessment).

Inclusion criteria:

• very good overall health (without chronic diseases);
• age: 30–55 years;
• there are no contraindications for whole body cryotherapy;
• written consent of the patient to participate in the study.

Exclusion criteria:

• consuming a lot of caffeine and / or alcohol (4 cups of coffee or 2 alcoholic drinks a day);
• change of diet during the project or in the month before;
• participation in other physical activities during the project or in the month before.

Characteristics of the participants

The experimental group consisted of 15 women and 15 men who underwent a series of whole-body cryotherapy treatments. The control group consisted of 15 women and 15 men - without intervention (Table 1).

**Table 1:** General characteristics of the respondents

Characteristics	WOMEN-CRYO n = 15	MEN-CRYO n = 15	WOMEN-CONTROL n = 15	MEN-CONTROL n = 15
Age [years]	38.47±5.80	35.87±7.83	35.87±7.48	30.20±4.46
Body height [cm]	169.40±5.60	179.67±9.30	167.73±7.40	182.73±6.92
Body mass [kg]	72.35±13.38	80.72±11.73	66.19±13.56	83.31±10.90
Body mass index [kg/m^2^]	25.22±4.65	25.06±3.52	23.48±4.27	25.01±3.61
Fat [% ]	30.47±6.43	19.08±6.55	25.75±6.07	15.17±5.60
Lean body mass [kg]	49.55±5.70	64.96±7.92	48.67±8.00	70.23±6.57
Total body water [kg]	36.28±4.17	47.57±5.80	35.62±5.86	51.42±4.81

### 2.2 Analysis of biochemical blood indices

For the analysis of blood biochemical parameters, venous blood was collected twice: Study 1: on the day of the commencement of whole body cryotherapy / from the control group; and Study 2: after a series of 20 cryotherapy sessions / from the control group (4 weeks).

The article "Effect of whole-body cryotherapy treatments on blood morphology and blood rheology: red blood cell deformability, red blood cell aggregation in healthy subjects" was published in 2023. Journal: Clin Hemorheol Microcirc.

Blood was collected from the subjects on an empty stomach in the morning from the antecubital, cephalic, or median vein into test tubes: with EDTA K2 (6 ml), with clotting activator (6 mL). The blood was collected by a qualified laboratory diagnostician, under the supervision of a physician, in accordance with the applicable standards.

Assessment of hematological parameters of the blood was done using the ABX MICROS 60 hematology analyzer (USA). The LORCA analyzer (Laser - Optical Rotational Cell Analyzer, RR Mechatronics, The Netherlands) was used to study erythrocyte aggregation and deformation. The obtained results are presented using two indicators: the elongation and aggregation index (EI and AI). The tests were performed according to the standard protocol: 30 minutes from the moment of collecting the material and at the temperature of 37°C [8, 13, 14].

### 2.3 Description of the intervention

Whole body cryotherapy (WBC) was performed at the Małopolska Rehabilitation Cryotherapy Center in Krakow. The temperature in the cryochamber is –120°C, and in the atrium: –60°C. Liquid nitrogen was used for cooling. Time of a single session according to the standard WBC protocol: 90 s (1 treatment); 120 s (2 treatments); 180 s (3–20 treatment). One treatment a day was performed (every day in the same time period, from 3:00 p.m. to 5:00 p.m.). A total of 20 treatments were performed and they were performed 5 times a week.

### 2.4 Statistical analysis

Descriptive statistics were determined: mean (x) as well as standard deviation (SD). The normality of distributions was verified with the Shapiro-Wilk test. Data distribution analysis was performed using parametric tests— the Student’s *t*-test for dependent samples within the group and the same test for independent samples performing comparisons within the groups. The applied tests verified two-sided hypotheses. The analyses were performed with the use of the Statistica 13 package (Tibco Software Inc., USA).

## 3 Results

After whole-body cryotherapy a statistically significant decrease in RBC, HGB, HCT, MCV, EI 0.30 and an increase in MCHC and EI 2.19–60.30 were observed in women, as well as a decrease in MCV, MCH, AI and an increase in PLT, EI 0.30–60.30, AMP, T1/2 in men. In people not receiving cryotherapy, a statistically significant decrease in EI 4.24–60.30 in both sexes and in AI in women, as well as an increase in T1/2 in women was observed (Table 2-3, Fig. 1).

**Table 2:** Intergroup comparisons of mean values of indicators - whole-body cryotherapy

Parameter	WOMEN-CRYO			MEN-CRYO		
	Study 1	Study 2	(p)	Study 1	Study 2	(p)
WBC (10^9^/L)	5,25±1,40	5,31±1,35	0,859	6,44±2,20	6,49±1,35	0,896
RBC (10^12^/L)	4,80±0,27	4,57±0,28	0,007*	5,22±0,34	5,18±0,32	0,441
HGB (g/dL)	13,39±0,80	12,88±0,73	0,014*	15,64±1,00	15,35±0,84	0,051
HCT (%)	40,54±2,50	38,35±2,20	0,003*	46,87±2,98	45,86±2,52	0,053
PLT (10^9^/L)	275,67±35,49	271,73±48,65	0,699	239,88±61,18	257,00±69,86	0,009*
MCV (fl)	84,40±4,03	84,00±4,16	0,028*	89,83±2,81	88,61±3,01	0,001*
MCH (pg)	27,94±1,61	28,25±1,60	0,090	29,97±0,95	29,62±1,01	0,005*
MCHC (g/dL)	33,05±0,65	33,60±0,42	0,013*	33,32±0,37	33,44±0,58	0,304
EI 0.30	0,05±0,02	0,02±0,01	0,001*	0,02±0,01	0,03±0,01	0,029*
EI 0.58	0,15±0,20	0,07±0,01	0,161	0,06±0,01	0,07±0,01	0,043*
EI 1.13	0,15±0,03	0,15±0,02	0,611	0,13±0,02	0,14±0,01	0,004*
EI 2.19	0,21±0,05	0,24±0,02	0,011*	0,21±0,03	0,23±0,01	0,000*
EI 4.24	0,26±0,07	0,33±0,02	0,001*	0,29±0,04	0,33±0,02	0,000*
EI 8.24	0,30±0,09	0,40±0,03	0,000*	0,34±0,05	0,40±0,02	0,000*
EI 15.98	0,36±0,09	0,47±0,02	0,000*	0,40±0,05	0,46±0,02	0,000*
EI 31.03	0,40±0,10	0,52±0,02	0,000*	0,44±0,06	0,51±0,02	0,000*
EI 60.30	0,42±0,09	0,56±0,02	0,000*	0,48±0,06	0,53±0,03	0,000*
AI (%)	58,28±8,04	58,96±7,51	0,688	58,56±6,29	55,45±6,58	0,035*
AMP (au)	21,62±4,06	21,91±2,07	0,742	21,36±3,41	24,46±2,33	0,000*
T1/2 (s)	2,81±1,03	2,75±1,11	0,800	2,68±0,73	3,129±0,92	0,024*

The article "Effect of whole-body cryotherapy treatments on blood morphology and blood rheology: red blood cell deformability, red blood cell aggregation in healthy subjects" was published in 2023. Journal: Clin Hemorheol Microcirc.

**Table 3:** Intergroup comparisons of mean values of indicators - without intervention

Parameter	WOMEN-CONTROL			MEN-CONTROL		
	Study 1	Study 2	(p)	Study 1	Study 2	(p)
WBC (10^9^/L)	5,91±1,91	5,26±0,95	0,189	5,29±1,05	5,17±1,46	0,675
RBC (10^12^/L)	4,32±0,26	4,36±0,18	0,402	5,08±0,33	5,07±0,35	0,734
HGB (g/dL)	12,51±1,29	12,53±1,21	0,880	15,24±0,97	15,18±1,16	0,691
HCT (%)	38,02±3,50	38,35±2,98	0,363	45,20±2,51	45,21±2,87	0,976
PLT (10^9^/L)	279,73±65,87	277,20±54,05	0,812	221,00±53,62	216,00±53,77	0,423
MCV (fl)	88,00±6,22	88,12±6,44	0,606	89,05±3,35	89,35±3,49	0,254
MCH (pg)	28,97±2,54	28,77±2,62	0,142	30,01±0,94	29,94±0,95	0,624
MCHC (g/dL)	32,23±2,24	32,61±0,99	0,555	33,71±0,80	33,53±0,83	0,302
EI 0.30	0,02±0,01	0,03±0,02	0,149	0,03±0,01	0,02±0,02	0,722
EI 0.58	0,08±0,02	0,09±0,03	0,187	0,09±0,01	0,14±0,18	0,307
EI 1.13	0,18±0,02	0,18±0,03	0,586	0,18±0,02	0,18±0,02	0,838
EI 2.19	0,29±0,02	0,28±0,02	0,100	0,29±0,02	0,29±0,02	0,161
EI 4.24	0,40±0,02	0,37±0,02	0,000*	0,40±0,02	0,38±0,03	0,009*
EI 8.24	0,48±0,01	0,44±0,03	0,000*	0,48±0,01	0,45±0,03	0,006*
EI 15.98	0,54±0,01	0,49±0,04	0,000*	0,54±0,01	0,51±0,04	0,009*
EI 31.03	0,58±0,01	0,53±0,04	0,000*	0,58±0,01	0,55±0,05	0,009*
EI 60.30	0,62±0,01	0,56±0,05	0,001*	0,62±0,01	0,58±0,05	0,005*
AI (%)	71,01±19,91	56,83±7,47	0,019*	52,87±7,54	55,35±51,18	0,170
AMP (au)	20,98±11,24	19,04±2,84	0,523	20,97±4,32	20,98±3,08	0,985
T1/2 (s)	1,96±1,29	3,00±0,98	0,028*	3,57±1,27	3,12±0,74	0,198

The article "Effect of whole-body cryotherapy treatments on blood morphology and blood rheology: red blood cell deformability, red blood cell aggregation in healthy subjects" was published in 2023. Journal: Clin Hemorheol Microcirc.

**Fig. 1:** Average values of EI at shear stress from 0.30 to 60.30 Pa in women and men receiving WBC and in women and men without intervention. [W-women; M-men; Cr-cryotherapy; C-control; 1-Study1; 2-Study2].

## 4 Discussion

This study is a continuation of our previous study with only men, in a smaller group, without a control group, and using only 10 cryotherapy treatments. As suspected, the conducted studies showed changes in the rheological properties of the blood in young healthy males undergoing WBC (increase RBC, HCT, PLT, decrease HGB, MCHC, MCH, MCV, AI) [14]. A review of the literature shows the lack of detailed data on the effect of systemic cryotherapy on the rheological properties of blood in healthy people.

The review of the data shows the lack of relevant and up-to-date data on the effect of systemic cryotherapy on the rheological properties of blood in healthy subjects.

Previous studies show that after several days of stimulation with cryogenic temperature, an increase in PLT, HGB, glucose and creatinine levels is observed [16, 17]. However, there are reports that show a decrease in RBC [18–22] and an increase in WBC [23, 24]. Some studies show no changes in RBC and / or WBC, presumably due to the low number of sessions [16, 19–21, 24]. Blatteis (1998) observed a decrease in WBC and RBC in healthy people after a series of treatments [25]. However, Banfi et al. (2008) showed a decrease in HBG concentration with a simultaneous increase in MCH and MCHC (30 seconds at 60°C and 2 min at –110°C) [18]. After the use of WBC in our volunteers, a statistically significant decrease in RBC, HGB, HCT, MCV and an increase in MCHC in women, and a decrease in MCV, MCH and an increase in PLT in men were observed. The conducted analysis showed no statistically significant changes in morphological parameters in patients without intervention.

Determining the elongation index and the aggregation index allows for the assessment of their rheological behavior. Rheological properties, such as aggregation which results in an increase in flow resistance, and deformation under the influence of a shear force leading to a decrease in flow resistance, are an important indicator of microcirculation, with erythrocytes occupying almost half the volume [26]. The phenomenon of RBC aggregation in whole blood is a physiological and fully reversible phenomenon, which at low shear rates of Shear Stress plays a very important role in blood flow and significantly increases blood viscosity [8]. The sites that are prone to the formation of RBC aggregates are mainly small blood vessels where shear rates are typically low. As a consequence, it causes a reduction in blood flow velocity, and even its complete inhibition, which unfortunately results in cell hypoxia [27]. After whole-body cryotherapy a statistically significant decrease in EI 0.30 and an increase in EI 2.19–60.30 were observed in women, as well as a decrease in AI and an increase in EI 0.30-60.30, AMP, T1/2 in men. In people not receiving cryotherapy, a statistically significant decrease in EI 4.24–60.30 in both sexes and in AI in women, as well as an increase in T1/2 in women was observed. The use of WBC has a stimulating effect by activating adaptive changes in the deformability of erythrocytes due general vasoconstriction. This form of therapy leads to increased pressure on the spleen and the release of erythrocytes into the bloodstream, which in turn results in differences in their deformability. Every day, under physiological conditions, 200–250 billion erythrocytes are broken down, and WBC can force red blood cells to break down faster. However, this requires further in-depth research.

The article "Effect of whole-body cryotherapy treatments on blood morphology and blood rheology: red blood cell deformability, red blood cell aggregation in healthy subjects" was published in 2023. Journal: Clin Hemorheol Microcirc.

To the best of our knowledge, this study is the first to evaluate the effects of white blood cells on blood rheology in men and women, including EI and AI levels. Earlier studies concern mainly sick people. In the past, we have noticed the influence of WBC on blood counts in various diseases: 10 treatments in women with rheumatoid arthritis (increase in RBC, HCT, AI and decrease in T½) [28], 20 treatments in women with multiple sclerosis (there was no significant effect on changes in blood count, rheology and biochemistry) [29]. Before and now, no pathological or harmful changes were observed after the use of WBC. Research should also continue to focus on healthy people, athletes, biological regeneration and the effects that the use of WBC may have in pathology-free conditions.

## 5 Conclusions

The use of whole-body cryotherapy causes changes in blood counts in various directions and has a positive effect on the rheological properties of blood in women and men - it increases the elongation index and reduces the aggregation index.

## Study limitation

This study is not without its limitations. An important aspect that could have affected trial results is the relatively small number of people in the experimental groups. The research should be continued in larger and more diverse groups of patients. In the future, the examined indicators should also be extended to include efficiency indicators.

## Data availability

All data generated or analyzed during this study are included in this published article.

## Conflicts of interest

All authors declare that they have no conflict of interest regarding the publication of this paper.

## Informed consent statement

Informed consent was obtained from all subjects involved in the study.

The article "Effect of whole-body cryotherapy treatments on blood morphology and blood rheology: red blood cell deformability, red blood cell aggregation in healthy subjects" was published in 2023. Journal: Clin Hemorheol Microcirc.

## Author contributions

Conceptualization, B.P.; data curation, S.P.; formal analysis, B.P. and S.P.; investigation, B.P. and S.P.; methodology, B.P., S.P., and A.T.; supervision, B.P., S.P., and A.T.; writing – original draft, B.P. and S.P.; writing – review and editing, B.P. and S.P. All authors have read and agreed to the published version of the manuscript.

## Funding

The publication is financed within the program of the Minister of Science and Higher Education in Poland under the name “Regional Excellence Initiative” in 2019–2022 (project number: 022/RID/2018/19) in the amount of PLN 11,919,908.
